The article "Protocatechuic aldehyde from Salvia miltiorrhiza exhibits an anti-inflammatory effect through inhibiting MAPK signalling pathway" was retracted in 2023. Reasons: errors in the images; unreliable results or conclusions; concerns about the images.

# Protocatechuic aldehyde from *Salvia miltiorrhiza* exhibits an anti-inflammatory effect through inhibiting MAPK signalling pathway

**DOI:** 10.1186/s12906-020-03090-4

**Published:** 2020-11-17

**Authors:** Shuang Wu, Qingyu Wang, Jinquan Wang, Baoyu Duan, Qihe Tang, Zhuojian Sun, Jinlong Han, Chenggang Shan, Zhifen Wang, Zhihui Hao

**Affiliations:** 1 Agricultural Bio-pharmaceutical Laboratory, Qingdao Agricultural University, Qingdao, 266109 China; 2 National Centre for Veterinary Drug Safety Evaluation, College of Veterinary Medicine, Agricultural University, Beijing, 100089 China; 3 College of Animal Medicine, Xinjiang Agricultural University, Wulumuqi, 830001 China; 4 College of Medical Technology, Shanghai University of Medical and Health Sciences, Shanghai, 201318 China; 5 Agricultural Products Processing Institute of Shandong Academy of Agricultural Sciences, Jinan, 250000 China; 6 Center of Research and Innovation of Chinese Traditional Veterinary Medicine, College of Veterinary Medicine, China Agricultural University, Beijing, 100089 China

**Keywords:** Protocatechuic aldehyde, *Salvia miltiorrhiza*, Anti-inflammatory, MAPK, NF-κB

## Abstract

**Background:**

The aerial parts of *Salvia miltiorrhiza*, which was considered to be the waste part and discarded during the root harvest, is rich in protocatechuic aldehyde (PAI). This study investigated the health-promoting effects of extracts and PAI from the aerial parts of *Salvia miltiorrhiza*, including its anti-inflammatory effects and the underlying mechanisms of action in vitro and in vivo.

**Method:**

Purification of the sample paste of *Salvia miltiorrhiza* was accomplished using HPLC analysis. TheMTT (Methylthiazolyldiphenyl-tetrazolium bromide) assay was employed to determine the cell viability. The production of inflammatory factors was detected by ELISA assays. The histopathological analysis was used to analyse the lungs and livers of mice treated with PAI. Western blot was performed to reveal the mechanism of PAI in anti-inflammatory.

**Results:**

The extracts and PAI from the aerial parts of *Salvia miltiorrhiza* inhibited TNF-α, IL-6 production and promoted the production of IL-10 in vivo in mice and in vitro in the macrophage cell line RAW264.7. NF-κB and MAPKs kinase phosphorylation were also suppressed by PAI in vivo and in vitro, indicating that PAI exhibited an anti-inflammatory effect.

**Conclusion:**

These findings suggest that the aerial parts of *Salvia miltiorrhiza* extract may serve as potential protective agents for inflammatory.

**Supplementary information:**

**Supplementary information** accompanies this paper at 10.1186/s12906-020-03090-4.

## Background

Sepsis is a systemic inflammatory response that can cause organ damages and acute lung injury, resulting in lethal consequences [1, 2]. Although modern intensive care practices have made great progress, the overall mortality for severe sepsis is still > 30%, with associated healthcare costs of $16.7 billion in the United States [3]. Furthermore, sepsis is also the leading cause of death from infectious diseases worldwide [4].

*Salvia miltiorrhiza* (Lamiaceae) roots, also known as Danshen in Chinese, has been used as one of the most popular traditional herbal medicines (TCM) in China and other East Asian countries [5]. *S. miltiorrhiza* Bunge is a perennial herb that has been widely used to treat cerebrovascular and cardiovascular diseases, hepatitis, kidney disease and menstrual disorders in traditional Chinese medicine [6–8]. Because of its various pharmacological properties, Danshen is one of the most important commercial herbs in China, which was consumed 5000–7000 tons every year [9–11].

The aerial parts of *S. miltiorrhiza* account for 60% of the whole plant. During the process of harvesting, the aerial parts are discarded as non-medicinal parts, causing a serious waste of resources and environmental pressure. Our study found that the aerial parts of *S. miltiorrhiza* are rich in phenolic acidsand revealed that can be utilized as reagents against inflammation. Our study not only can improve economic growth, but also help reduce resource waste and pollution.

Both the aerial parts and underground parts of *Salvia miltiorrhiza* contain a large amount of phenolic acids, and the content of the underground parts is higher than that of the aerial parts. The difference between the two parts is that the root of *Salvia miltiorrhiza* contains a large amount of tanshinone, which does not exist in the aerial parts. Both have the effects of improving cardiovascular, promoting tissue repair, antibacterial and anti-inflammatory.

Protocatechuic aldehyde (PAI) (3,4-dihydroxy-benzaldehyde), one of the active water-soluble phenolic compounds derived from Danshen [12], has been proved to have multiple therapeutic effects. It has been used to protect against isoproterenol-induced cardiac hypertrophy via JAK2/STAT3 inhibition as well as inhibiting hyaluronan production in fibroblasts derived from Graves orbitopathy patients [5, 13]. PAI also inhibited TNF-α-induced fibronectin expression in human umbilical vein endothelial cells via the JNK and NF-κB pathways [14]. In addition, PAI has been reported to prevent experimental pulmonary fibrosis by modulating the high-mobility group box protein 1 (HMGB1) with the receptor for advanced glycation end-products (RAGE) [15]. Cisplatin-induced decline of renal function can also be prevented by PAI [16].

However, many of the molecular components mediating the anti-inflammatory effects of PAI have not been fully explored. Therefore, in this study, we aim to investigate the anti-inflammatory effects of PAI both in vivo and in vitro.

## Methods

### Chemicals and reagents

Ursolic acid, salvianolic acid A, salvianolic acid B, Danshensu, and Protocatechuic aldehyde (purity > 99%) were supplied by the National Institute for the Control of Pharmaceutical and Biological Products (Beijing, China). Acetonitrile (ACN) used in high performance liquid chromatography (HPLC) was purchased from Fisher Scientific (Pittsburgh, PA. USA). Phosphoric acid and ethanol (analytical grade) were obtained from Beijing Beihua Fine Chemicals (Beijing, China). Deionized water was purified by the Milli-Q System (Millipore, Bedford, MA, USA). Penicillin, streptomycin, and fetal bovine serum (FBS) were purchased from Hyclone (Logan, UT, USA). Lipopolysaccharide (LPS) and Dulbecco’s modified Eagle’s medium (DMEM) were purchased from Gibco BRL (Grand Island, NY, USA). 3-(4,5- dimethylthiazol − 2-yl)-2,5-diphenyltetrazolium bromide (MTT), 2,3,5-triphenyl tetrazolium chloride (TTC), and Trypan blue dye were obtained from Sigma (St. Louis, MO, USA). All other chemicals and solvents used were purchased from Sinopharm Chemical (Shanghai, China) and all of them were of analytical grade or better.

### Experimental animals

C57 mice of equal sexes (18–22 g) were obtained from Daren Fucheng (Qingdao, China). The mice were maintained at 25 ± 2 °C with free access to food and water as prescribed by the Guidelines of Experimental Animal Care issued by the Animal Welfare and Research Ethics Committee at Qingdao Agriculture University.

### Plant materials and sample preparation

The aerial parts of *S. miltiorrhiza* were purchased from Department of Medicinal Plants, Shandong Academy of Agricultural Sciences. They were collected in late fall, dried to a constant weight at 35 °C, and grounded to a fine powder. The powder samples (2 kg) were refluxed twice in 75% ethanol for 1.5 h each time and filtered using solvent filter (Fei Teng, Tianjing, China). The filtrate was concentrated under reduced pressure at 60 °C to a paste with a relative density ranging from 1.18 to 1.22. After the centrifugal removal of chlorophyll, the ethanol was recovered under reduced pressure. The remainders of the sample were concentrated to a thick paste and vacuum dried. The components of the sample paste were analysed quantitatively using HPLC. The resulting extract was partitioned sequentially with petroleum ether, chloroform, ethyl acetate, and n-butanol, followed by freeze drying to yield the petroleum ether fraction (extract A), the chloroform fraction (extract B), the ethyl acetate fraction (extract C), the n-butanol fraction (extract D).

### HPLC analysis

Purification of the sample paste was accomplished using an Agilent 1260 HPLC system (Agilent Technologies, Santa Clara, CA, USA). The separation was performed with a 250 × 4.6 mm, 5 μm, Ultrasphere C18 column (Alltech, Deerfield, IL, USA). Distilled water (solvent A) and 0.2% phosphoric acid (solvent B) were used as the mobile phase at 0.8 mL/min, along with a column temperature of 25°Cand a detector wavelength of 285 nm. The injection volume was 10 μL. Analytes were eluted using a gradient as follows: 0–5 min, 10–15% A; 5–12 min, 15–30% A; 12–20 min, 30–45% A; 20–25 min, 45–15% A; 25–30 min, 15%–10% A.

For the sample assay, 10 μL of PAI solution was injected. The assay was repeated three times. All solutions were filtered through Millex 0.45-mm nylon membrane syringe filters (Millipore Co., Bedford, MA, USA) before use.

### Survival rate

C57 mice were divided into 7 groups of 10 mice each as follows: blank group, LPS group, administration group (1 μg/mL) (extract A, extract B, extract C, extract D), dexamethasone (200 μg/mL). The sepsis model was established by injecting the same volume of LPS (100 ng/mL) into each group, except that the blank group was given normal saline. Gastric administration for the assigned groups started at 1-h post injection. The LPS group and the blank group were given normal saline of equal volume. The mortality rate of mice was calculated 7-day post injection.

### Purification

The extract having a high survival rate effect in mice assay was subjected to polyamide column chromatography, followed by freeze drying. The obtained substance was dissolved in ethanol and detected by HPLC. The purified substance was diluted with ethanol to different concentrations for the study of the anti-inflammatory activities and underlying mechanisms of action.

### Cell culture

The murine macrophage cell line RAW264.7 (ATCC TIB-71) was seeded and cultured in 96-well tissue culture plates (Costar, Cambridge, MA, USA) in DMEM medium with 10% FBS, in a humidified atmosphere (37 °C, 5% CO_2_)_._ Routine cell viability measured by Trypan blue dye indicated over 80% viability [17].

### The measurement of cell viability

Cell viability was determined using a commercial MTT assay kit (Jiancheng Bioengineering Institute, Nanjing, China) and the experimental procedures were suggested by the manufacturer. RAW264.7 cells were seeded at 2 × 10^4^ cells/well in a 96-well plate and incubated for 24 h. Aliquots of different density purification were added with four replicates, and the incubation continued for another 24 h. 4 h prior to the end of incubation, 10 μL of MTT solution (2 mg/ml) was added to each well. Once the incubation period was over, 150 μL of DMSO solution were added to each well. After 15 min of incubation, the absorbance was read at wavelengths of 490 nm.

### Animals and treatments

C57 mice were divided into 5 groups of 10 mice each: (1) Control (saline only); (2) LPS (100 ng/kg) intraperitoneal (ip) once; (3) PAI (0.25, 0.5 and 1 μΜ) intraperitoneal (ip) once. After 48 h, mice were euthanized by CO_2_ asphyxiation. At the end of the experimental period, the mice were sacrificed according to the protocol approved by the animal care and use committee. Blood, heart, liver, spleen and lungs were collected and prepared for hematoxylin and eosin (H&E) staining, Western blotting, and ELISA.

### Histochemical assay

The heart, liver, spleen, lung and kidney tissues were fixed in 4% paraformaldehyde and embedded in paraffin. The paraffin embedded tissue samples were sectioned into 5 μm thickness and stained with hematoxylin and eosin [18].

### ELISA assays

TNF-α, IL-6, and IL-10 levels were measured using commercial ELISA kits according to the manufacturer’s instructions (Tumor Necrosis Factor-α Assay Kit; Interleukin-6 Assay Kit; Interleukin-10 Assay Kit; Jiancheng Bioengineering Institute, Nanjing, China).

### Western blot assay

Tissue samples for protein assays were quickly frozen in liquid nitrogen and pulverized with a mortar and pestle. Tissue powder was added to 1.5 mL Eppendorf tubes and solubilized in RIPA buffer containing protease inhibitors (Bio-Rad, Hercules, CA, USA). 30–80 μg of total protein based on the measurements using a Bradford assay (Bio-Rad, Hercules, CA, USA) were visualized using 10% SDS-PAGE minigels (Jiancheng Bioengineering Institute, Nanjing, China). The gels were transferred onto nitrocellulose membranes using standard procedures [19]. Gel bands were scanned and quantified with the Gelpro 3.0 software (Jiancheng Bioengineering Institute, Nanjing, China).

### Statistical analysis

All experiments were repeated at least three times. Results were calculated as mean ± standard deviation (SD) and analyzed using GraphPad Prism 5.0. Comparisons between experimental groups were conducted by using one-way ANOVA, whereas multiple comparisons were made by using the LSD method. Statistical signifificance was defifined as *P < 0.05 .

## Results

### HPLC analysis

The extracts of aerial parts of *S. miltiorrhiza* mainly contained ursolic acid, salvianolic acid A, salvianolic acid B, protocatechuic aldehyde, Danshensu and other substances (Fig. 1a, b, and Supplementary figure 1).

**Fig. 1:** High-performance liquid chromatography chromatograms of *S. miltiorrhiza*’s sample paste. The sample was taken from the aerial part of *Salvia miltiorrhiza* and mainly contains Ursolic acid, Salvianolic acid A, Salvianolic acid B, Protocatechuic aldehyde, Danshensu five phenolic substances. After purification with chloroform, it mainly contains protocatechuic aldehyde. **a** Standard mixture, **b** Purification. **c** The aerial portions’ extracts of *S. miltiorrhiza*. Ursolic acid (1), Salvianolic acid A (2), Salvianolic acid B (3), Protocatechuic aldehyde (4), Danshensu (5)

### Survival rate

The survival rate of control group was set as 100%. Compared with the LPS group, the mice in extract B group had the highest survival rate, while the extract D group had the lowest survival rate. Survival rate of extract C is similar to that of extract A. The survival rate of extract B is almost 1.5 times that of extract A / C. These results suggested that the extract B group had a good anti-inflammatory effect (Supplementary figure 2).

### Purification

The extract B, which has better anti-inflammatory effect than other fractions, was dilute with ethanol and purified it with D101 macroporous adsorption resin. The purified extract B mainly contained protocatechuic aldehyde. The purified PAI was used to study its anti-inflammatory activity and mechanism of action in the later stage (Fig. 1a and c).

### Cell viability after PAI treatment

We first tested the effects of PAI on macrophage viability in cell culture. The cell viability was significantly upregulated at 0.25, 0.5, and 1 μM of PAI in comparison to the LPS group (Fig. 2).

**Fig. 2:** Effects of protocatechuic aldehyde on cell viability in RAW 264.7 cells. The cell viability was measured by MTT method, and the cells were 6th-generation RAW264.7 cells. Data are presented as mean ± SD (*n* = 4). #*p* < 0.05, ##*p* < 0.01, ###*p* < 0.001 vs controls. *p < 0.05, **p < 0.01, ***p < 0.001 vs LPS group

### Histopathological changes

The lungs and livers of LPS-challenged mice displayed signs of edema and interstitial inflammation. The effect in lung tissue is more obvious. In the LPS group, inflammatory cells infiltrated into the lung tissue, the amount of bleeding increased at the bleeding points and, and the lungs had obvious plasma exudation and showed a transparent membrane, and the pulmonary edema was obvious. The livers showed increased inflammatory cell infiltration as well as moderate portal inflammation and hepatocellular necrosis. However, PAI attenuated these pathological changes and high-dosages work better. The results are consistent with the literature description [13] (Fig. 3a-d).

**Fig. 3:** Immunodetection of inflammation markers of mice treated with protocatechuic aldehyde. Sampling from C57 mice, Immunodetection was performed with two pro-inflammatory cytokines (IL-6 and TNF-α) of lung. Histological micrographs of liver and lung. Representative sections for ten mice per group are shown. Scale bar = 200 μm. **a** Histological micrographs of liver. **b** Histological micrographs of lung. **c** Histological micrographs of lung stained with IL-10 antibody. **d** Histological micrographs of lung stained with TNF-α antibody. Arrows: obvious inflammatory cells

### PAI reduces TNF-α and IL-6 level while increases IL-10 expression in vivo and vitro

For mice that were challenged with LPS, the level TNF-α and IL-6was increased both in vivo and in vitro as expected (Fig. 4 and Supplementary figure 3, 4, and 5). Simultaneous administration of PAI resulted in an increase in IL-10 expression in comparison to the LPS group (Fig. 4 and Supplementary figure 5).

**Fig. 4:** The effect of Protocatechuic aldehyde on IL-6, IL-10, and TNF-α levels in vitro. Sampling from C57 mice, two pro-inflammatory cytokines (IL-6 and TNF-α), and one anti-inflammatory cytokine (IL-10) were measured at the mRNA and/or protein levels and data were presented as percentages of WT values. Eight to five (mRNA) or five (protein) mice per group. Data are presented as mean ± SD (*n* = 4). #*P* < 0.05, ##*P* < 0.01, ###*P* < 0.001 vs LPS. *P < 0.05, **P < 0.01, ***P < 0.01 vs controls group. $*P* < 0.05, $$*P* < 0.01, $$$*P* < 0.01 LPS vs controls group

### The effects of PAI on NF-κB and MAPK signalling

The NF-κB and MAPK pathways cause the activation of ERK, p38 and JNK in response to septic shock in most cell types. As expected, LPS administration resulted in increased phosphorylation of p38, ERK, JNK, IκB and NF-κB p65 significantly both in vivo and in vitro. PAI treatment significantly suppressed p38, ERK and JNK phosphorylation in a dose-dependent manner (Figs. 5 and 6).

**Fig. 5:** The effects of Protocatechuic aldehyde on NF-κB and MAPK pathways in vivo*.* Sampling from C57 mice, mainly two signal pathways (NF-κB and MAPK pathways) were detected. Effects of protocatechuic aldehyde on the expression of ERK/P38/JNK protein in the MAPK pathway of RAW264.7 cells. Effects of protocatechuic aldehyde on the expression of IκB / P65 protein in the NF-κB pathway of RAW264.7 cells. **a** The effects on MAPK pathways in vivo. **b** The effects on NF-κB pathways in vivo. Data are presented as mean ± SD (*n* = 4). #*P* < 0.05, ##*P* < 0.01, ###*P* < 0.001 vs LPS. *P < 0.05, **P < 0.01, ***P < 0.01 vs controls group

**Fig. 6:** The effects of Protocatechuic aldehyde on NF-κB and MAPK pathways in vitro*.* Sampling from C57 mice, mainly two signal paths (NF-κB and MAPK pathways) were detected. Effects of protocatechuic aldehyde on the expression of ERK / P38 / JNK protein in the MAPK pathway of RAW264.7 cells. Effects of protocatechuic aldehyde on the expression of IκB / P65 protein in the NF-κB pathway of RAW264.7 cells. **a** The effects on MAPK pathways in vitro. **b** The effects on NF-κB pathways in vitro. Data are presented as mean ± SD (*n* = 4). #*P* < 0.05, ##*P* < 0.01, ###*P* < 0.001 vs LPS. *P < 0.05, **P < 0.01, ***P < 0.01 vs controls group

## Discussion

The chemicals from the root part of S. miltiorrhiza has been studied extensively for its bioactivity in the literature in recent years, but there is few reports on the bioactivity of extract from its aerial parts [7]. We carried out research on extracting protocatechuic aldehyde from the aerial part of S. miltiorrhiza, and explored its main medicinal effects. Although the effects of polysaccharides and some TCM monomers on inflammatory factors have been studied, the effects of PAI on inflammatory factors remain unknown [20, 21]. In the present study, we found that the administration of PAI improved the survival rate of mice and cells and attenuated the LPS induced acute phase response in an LPS mice model. Besides, some tissue sections show that PAI can reduce liver and lung damage.

Some studies have also found that lethality from sepsis or septic shock is primarily associated with the high levels of serum TNF-α, IL-6 [12, 15]. The literatures indicate that the over-secretion of proinflammatory cytokines aggravates sepsis progression, and TNF-α and IL-6 are the most important early proinflammatory cytokines that are secreted within a few minutes after an endotoxin challenge [15]. We show PAI suppressed the secretion of the proinflammatory cytokines TNF-α and IL-6 which contribute to the septic shock induced by LPS. Importantly, PAI also elevated the immunosuppressive cytokine IL-10 level (see Fig. 1 and Fig. 2). These endogenous inflammatory mediators modulate the pathophysiology of the systemic inflammatory response syndrome associated with sepsis. In summary, our results indicate that PAI can regulate some inflammatory factors in RAW264.7 cells and mice.

Some studies have shown that theexpression of inflammatory factors can be increased by MAPK and NF-κB pathways. MAPK is an important kinase in the redox signal transduction of microglia. It regulates the gene expression of proinflammatory factors, chemokines, and enzymes. The MAPK pathway includes three key molecules, ERK, P38, and JNK. Among them, P38 and JNK, as stress-activated kinases, play a key role in cell stress, apoptosis and inflammation, and participate in the occurrence of many cases. The ERK pathway mainly plays a role in promoting cell survival and inhibiting programmed cell death, and plays a protective role in some pathological processes. It has been reported before that the transcriptional activator NF-κB and MAPK arekey factors in septic shock as they exert a range of versatile functions [22, 23]. We found that PAI administration is associated with the alterations in MAPK and NF-κB signaling. Our in vitro and in vivo results indicated a significant protective effect for PAI. We found that PAI inhibited the increases in NF-κB activation and MAPK pathway expression in septic shock, indicating these two factors have an essential role in the septic shock attenuation by PAI.

## Conclusion

Together, we demonstrated that PAI exhibited a protective effect by modulating the expression of inflammatory cytokines in vitro and in vivo*.* PAI exerts its anti-inflammatory activities by modulating the phosphorylation of IκB-α and p65 and inhibiting the phosphorylation of p38, ERK and JNK in a dose-dependent manner.

## Supplementary information

**Additional file 1.**

## Data Availability

Not applicable.

## Abbreviations

PAI: Protocatechuic aldehyde
HMGB1: High-mobility group box protein 1
RAGE: Receptor for advanced glycation end-products
HPLC: High performance liquid chromatography
FBS: Fetal bovine serum
LPS: Lipopolysaccharide
DMEM: Dulbecco’s modified Eagle’s medium
